The article "Association between the Predicted Value of APACHE IV Scores and Intensive Care Unit Mortality: A Secondary Analysis Based on EICU Dataset" was retracted in 2023. Reasons: signs of a paper mill; suspected computer-generated content; unreliable results or conclusions; concerns about the data.

# Association between the Predicted Value of APACHE IV Scores and Intensive Care Unit Mortality: A Secondary Analysis Based on EICU Dataset

**DOI:** 10.1155/2022/9151925

**Published:** 2022-04-06

**Authors:** Yuan Xu, Sheng Chao, Yulin Niu

**Affiliations:** Department of Organ Transplantation, Affiliated Hospital of Guizhou Medical University, Guiyang 550004, China

## Abstract

**Objective:**

The evidence regarding the relationship between Acute Physiological and Chronic Health Assessment (APACHE) IV scores and emergency intensive care unit (EICU) mortality in patients following organ transplantation remains controversial. The purpose of this study was to investigate the relationship between APACHE IV score and EICU mortality.

**Methods:**

Data from 391 American men and women admitted to the EICU after undergoing organ transplants including heart, bone marrow, liver, kidney, lung, and pancreas in the United States. We used this data to analyze the relationship between APACHE IV scores and in-hospital mortality in the postoperative EICU. The primary endpoint was ICU hospitalization mortality after organ transplantation. The entire study data was extracted from the EICU database and uploaded to the DataDryad website.

**Results:**

Interaction tests indicate age, respiratory failure, and hormone use can modify the association between APACHE IV and EICU mortality. A stronger association of APACHE and mortality can be observed at <60 years old, no respiratory failure, and no use of hormones. In contrast, there was no association between respiratory failure, hormone use, APACHE, and ICU mortality in patients over 60 years of age.

**Conclusion:**

When using the APACHE score for risk stratification of critically ill patients after transplantation, the patient's age, respiratory failure, and use of hormones should be taken into account.

## 1. Introduction

As an indicator to evaluate the severity of patients, Acute Physiological and Chronic Health Assessment (APACHE) IV score is often used to evaluate the prognosis of critically ill patients in intensive care unit (ICU) [1–4]. The score is updated regularly in a database in North America. In the past, we used APACHE II/III for the assessment, but this version proved to overestimate the mortality rate [1, 5]. Most studies have suggested that APACHE IV has a good ability to discriminate and calibrate hospital mortality predictions, but there are few reports of significant differences among patients admitted to the emergency ICU (EICU) after organ transplantation [6–8]. Previous studies have shown that APACHE IV can better predict the severity of disease in EICU patients with acute trauma [3]. Due to the complexity of the disease, mortality after admission to the EICU is usually related to age, prior chronic disease status, and the presence or absence of complicated organ failure [9]. APACHE IV predicted mortality showed excellent differences in predicting in-hospital mortality as evaluated by area under curves (AUC) [10–12]. However, previous studies investigated the correlation between the APACHE IV score and EICU mortality and reported the opposite result. Some studies believe that SAPS3 and APACHE II scores perform poorly in kidney transplant patients and overestimate mortality [13]. We speculate that these conflicting results may come from differences in the study population and adjustment of covariates.

Therefore, we conducted a secondary analysis based on Philips-EICU database tables. This was a multicenter cohort study to investigate the correlation between the APACHE IV score of critically ill patients after organ transplantation and EICU mortality.

## 2. Methods

### 2.1. Data Source

Analysis was released for use in specific database tables from the EICU website (http://links.lww.com/CCM/F753). In order to allay potential privacy concerns, 391 organ transplant cases from the EICU were nonselectively collected, and in this study, participants' identity information was encoded as an untraceable code. Clinical data was stored by an electronic data acquisition system. Following a web-based training course and the Protection of Human Study Participants exam (No. 36208651), we obtained a license to extract data from the EICU-CRD. Because the study was designed retrospectively and anonymous data was analyzed, informed consent of the participants was not required.

### 2.2. Study Population

This study is a multicenter retrospective cohort study. Initially, 200859 participants were initially involved in this study; 200468 participants were subsequently excluded from this study, leaving 391 cases for the final data analysis (Figure 1). The start time and end time of the clinical data collection for these involving participants were 2014-2020, respectively. All clinical procedures in this study follow the guide.

Inclusion criteria included are the following: (1) patients admitted to EICU after organ transplantation; (2) patients who died before admission to EICU were excluded.

Exclusion criteria included are the following: (1) no APACHE IV score and (2) lack of death information.

### 2.3. Variables

#### 2.3.1. APACHE Rating

We obtained the APACHE IV score information at baseline and recorded it as a continuous variable. The detailed process for defining the APACHE IV score is described on the EICU official website (http://links.lww.com/CCM/F753). In addition to the specific APACHE IV score, the EICU download data also provides the specific variable parameters used to calculate APACHE IV.

#### 2.3.2. EICU Mortality

The outcome variable we were interested in was EICU mortality (dichotomy: 1: survival and 0: death).

#### 2.3.3. Covariates

The covariates involved in this study were selected based on our clinical experience and risk factors reported in the literature, and the study was concerned with death in the EICU. The APACHE IV score grouping is based on the data of 391 cases of organ transplant patients who have died in EICU. According to the above principles, the following variables are used as covariates: (1) continuous variables: age, body mass index (BMI), hemoglobin, platelet count, and APACHE IV score; (2) categorical variables: gender, use of immune drugs, chronic obstructive pulmonary disease (COPD), hypertension, sepsis, and glucocorticoids. Patients were divided into two groups: the APACHE IV score ≥ 70 group and <70 group according to Table 1.

### 2.4. Statistical Analysis

Continuous variables were expressed as mean ± standard deviation (SD) (Gaussian distribution) or median (range) (skewed distribution). Categorical variables were reported as number (%). We used *χ*^2^ (categorical variables), one-way ANOVA test (normal distribution), or Kruskal-Wallis H test (skewed distribution) to test for differences among different APACHE IV scores. Univariate and multivariate binary logistic regression models were used to test the connection between APACHE IV score and EICU mortality with three distinct models. In addition, threshold saturation effects were used to identify clinical inflection points in the APACHE IV score that might lead to different outcomes. The hierarchical binary logistic regression model was used for subgroup analysis. For continuous variables, we first converted them to categorical variables based on clinical cut-off points or dichotomies and then conducted interaction tests. The effect modification of subgroup indicators was tested, and then, the likelihood ratio was tested. To test the robustness of our results, we performed a sensitivity analysis.

Modeling was performed with the statistical software packages R (http://www.R-project.org, The R Foundation) and EmpowerStats (http://empowerstats.com, X&Y Solutions, Inc, Boston, MA). *P* values of less than 0.05 (two-sided) were considered statistically significant.

## 3. Results

### 3.1. Baseline Characteristics of Participants

The baseline characteristics of these participants are listed in Table 2. The mean age was 56.34 ± 12.42 years old, and the male was 59.64%. The mortality rate was 4.859% (19/391). There were no statistically significant differences in APACHE IV score (dichotomous) between groups, gender, sepsis, immunosuppressant use, history of COPD, and glucocorticoid use (*P* > 0.05). Continuous variables such as BMI, hemoglobin, and platelet count were significantly increased in patients with APACHE IV ≥ 70 compared to the APACHE IV < 70 group. The combination of respiratory failure among the categorical variables was significantly related to APACHE IV score and EICU death of patients.

### 3.2. The Results of Multivariate Analyses Using a Binary Logistic Regression Model

Unadjusted model results showed that the risk of death increased by 3% for each 1-point increase in score (OR, 1.03; 95% CI, 1.02-1.05; and *P* < 0.05). The same results were observed in both unadjusted and fully adjusted models. Thus, the APACHE IV score was positively associated with death with or without adjustment for covariates (Table 3).

### 3.3. The Results of Subgroup Analyses

In this study, we used variables such as gender, age, respiratory failure, sepsis, use of hormones, use of tacrolimus, and use of mycophenolate as potential effect-modifying factors. Through interaction test, we explored which factors might modify the association between APACHE IV and death (Table 4). In that case, age was used as a continuous variable and was grouped according to age 60. The results showed that gender, sepsis, tacrolimus, and mycophenolate did not modify the APACHE IV-death relationship (*P* value for interaction >0.05). But age, respiratory failure, and hormone use modified the association (*P* value for interaction <0.05). For age, in those younger than 60 years, we observed that increased APACHE IV scores were associated with mortality (OR, 1.05 and 95% CI, 1.02-1.09). In those older than 60 years, the relationship was not seen (OR, 1.00 and 95% CI, 0.97-1.04). For patients with combined respiratory failure, the association between APACHE IV score and death was not significant. However, for patients without respiratory failure, a higher APACHE IV was associated with an increased risk of death after admission to the ICU (OR, 1.05 and 95% CI, 1.02-1.08). In patients with respiratory failure, no such association was seen (OR, 1.00 and 95% CI, 0.97-1.03). For those glucocorticoids, in individuals who did not take glucocorticoids, an APACHE IV-death relationship was observed (OR, 1.05 and 95% CI, 1.02-1.08). In glucocorticoid users, no difference in the relationship was found (OR, 0.99 and 95% CI, 0.96-1.03).

## 4. Discussion

In this observational retrospective cohort study, we examined the association of APACHE IV score with EICU mortality in severe patients after organ transplantation. Our findings suggested that the increases in APACHE IV score were correlated with a significantly increased risk of death. This was similar to the results of many studies. Based on data collected from patients at 104 intensive or coronary care units in 45 hospitals, Zimmerman et al. reported that APACHE IV has good identification and calibration ability for the prediction of hospital mortality [1, 14]. Lee et al. [2] used patients who had undergone living donor or deceased donor liver transplantation were admitted to the surgical ICU as the study population and obtained similar results. Besides, Tian et al. [15] showed that the APACHE II score on day 3 of hospitalization was the best biomarker to predict prognosis in ICU patients. However, our results differ from the conclusions of existing studies. Freitas et al. reported that among organ transplant patients requiring ICU management, the SAPS3 and APACHE IV scores performed poorly in this population and overestimated mortality [16]. By comprehensive consideration of factors such as study design, population, we speculate that the causes of inconsistent results may be related to the factors.

Most existing studies assessing the risk of death from organ transplantation have focused on a single organ transplant and looked at fewer variables [17–20]. Our study included patients with severe organ transplantation in the EICU, including heart transplantation, bone marrow transplantation, liver transplantation, kidney transplantation, lung transplantation, and a few pancreas transplantation patients, and involved a more comprehensive type of organ transplantation. We also found that hormone use may act as an interacting factor that attenuates the predictive effect of APACHE IV on patient death. In contrast, factors such as immunosuppressant use and sepsis/respiratory failure, previously considered in clinical experience, did not influence the risk of occurrence of death in patients assessed by APACHE IV in this study. Lissauer et al. [21] showed that patients with high APACHE III scores in ICU readmission were more likely to have a history of immunosuppression. There are also differences in correlation with reported mortality and infection in the ICU after liver transplantation, as well as prolonged ICU stay [22].

Our study has some strengths, and we listed then as follows. (1) Interaction analysis is used, which can help us better understand the correlation between APACHE score and death. (2) We used multiple regression equations and sensitivity analysis (both for APACHE as a continuous variable and as a categorical variable) to ensure robustness. (3) We adopted a strict adjustment strategy to minimize the influence of confounding factors. Our design provides higher evidence level than the previous design. To our knowledge, this is the first time we have observed a link between APACHE IV score and EICU mortality in severe patients after organ transplantation. Most covariates have complete information, with a few missing. In this study, we tested the robustness of the results through a series of sensitivity analyses (target independent variable transformation, subgroup analysis, log-likelihood ratio test, etc.) to ensure the reliability of the results.

Our research has the following shortcomings and needs attention: first, our findings can be generalized to severe patients after organ transplantation only; second, as in all observational studies, even though known potential confounders factors were controlled for, there might still have been unmeasured confounders; third, our study population is from the United States. Therefore, it has geographical and national limitations. If applied to other populations or countries, the results need to be interpreted with greater caution.

In conclusion, we found that age, respiratory failure, and glucocorticoids can modify the APACHE IV-death relationship. These three factors should be taken into account when using the APACHE IV-score for risk stratification of critically ill patients after transplantation.

## Figures and Tables

**Figure 1:** Participant screening flow chart.

**Table 1:** Threshold saturation effect.

Outcome	Death in EICU ward
The model I	
Linear effect	1.03 (1.02, 1.05) 0.0002
The model II	
Fold point (K)	70
<K segment effect 1	1.00 (0.96, 1.04) 0.9925
>K segment effect 2	1.05 (1.02, 1.08) 0.0003
The effect of 2 is not equal to 1	1.05 (0.99, 1.11) 0.0915
Predicted value of the equation at the break point	-3.80 (-4.81, -2.79)

Data in table: *β* (95% CI) *P* value/OR (95% CI) *P* value. Outcome variables: death in ICU ward; exposure variables: acute physiology score (IV); adjust the variable: none.

**Table 2:** Baseline characteristics of participants.

	APACHE IV < 70 group (*n* = 283)	APACHE IV ≥ 70 group (*n* = 108)	Standardize diff.	*P* value	*P* value^∗^
Age (years)	56.23 ± 12.96	55.90 ± 11.18	0.03 (-0.19, 0.25)	0.815	0.456
BMI	27.86 ± 8.28	31.39 ± 21.10	0.22 (-0.00, 0.44)	0.018	0.101
HB	10.75 ± 2.40	10.07 ± 2.14	0.30 (0.08, 0.52)	0.010	0.005
PLT	182.14 ± 99.24	125.26 ± 80.92	0.63 (0.40, 0.85)	<0.001	<0.001
Male/female	171/112	65/43	0.00 (-0.22, 0.23)	0.966	
Death in ICU ward			0.28 (0.06, 0.50)	0.004	-
Alive	277 (97.88)	99 (91.67)			
Death	6 (2.12)	9 (8.33)			
Acute respiratory failure			0.47 (0.25, 0.70)	<0.001	-
No	236 (83.39)	68 (62.96)			
Yes	47 (16.61)	40 (37.04)			
COPD			0.09 (-0.13, 0.31)	0.434	-
No	267 (94.35)	104 (96.30)			
Yes	16 (5.65)	4 (3.70)			
Drug			0.34 (0.12, 0.56)	0.068	-
Tacrolimus	111 (39.22)	32 (29.63)			
Mycophenolate mofetil	72 (25.44)	41 (37.96)			
Sirolimus	10 (3.53)	3 (2.78)			
Athers	33 (11.66)	7 (6.48)			
Unknown	57 (20.14)	25 (23.15)			
Sepsis			0.16 (-0.06, 0.38)	0.143	-
No	238 (84.10)	84 (77.78)			
Yes	45 (15.90)	24 (22.22)			
Glucocorticoid			0.05 (-0.17, 0.28)	0.632	-
No	170 (60.07)	62 (57.41)			
Yes	113 (39.93)	46 (42.59)			
Transplant type			0.50 (0.25, 0.74)	0.002	-
Heart transplant	43 (19.91)	19 (20.21)			
Bone marrow transplant	9 (4.17)	2 (2.13)			
Liver transplant	45 (20.83)	26 (27.66)			
Kidney transplant	113 (52.31)	41 (43.62)			
Lung transplant	0 (0.00)	6 (6.38)			
Pancreas transplantation	6 (2.78)	0 (0.00)			

Data were mean ± SD or *n* (%). APACHE: Acute Physiological and Chronic Health Assessment; BMI: body mass index; HB: hemoglobin; PLT: platelet; ICU: intensive care unit; COPD: chronic obstructive pulmonary disease. *P* value^∗^: for continuous variables, it is obtained by Kruskal-Wallis rank sum test. If the count variable has a theoretical number < 10, it is obtained by Fisher's exact probability test.

**Table 3:** Multivariate analyses of the effect of APACHE IV score on death in ICU.

Exposure	Nonadjusted			Adjust I			Adjust II		
	OR	95% CI	*P* value	OR	95% CI	*P* value	OR	95% CI	*P* value
APACHE IV	1.03	1.02, 1.05	0.0002	1.03	1.02, 1.05	0.0002	1.03	1.01, 1.05	0.0089
APACHE IV									
<70	1.0			1.0			1.0		
≥70	4.20	1.46, 12.09	0.0079	4.24	1.47, 12.25	0.007	3.77	0.95, 14.95	0.0588

Outcome variables: death in ICU ward; nonadjusted model adjust for: none; adjust I model: adjust for gender and age (years); adjust II model: adjust for gender and age (years), BMI, hemoglobin, platelet count, acute respiratory failure, whether to merge COPD, whether to be combined with hypertension, whether it is sepsis, and whether glucocorticoids were used.

**Table 4:** Effect of APACHE IV score on death in ICU ward subgroups.

Characteristic	Number of participants	Effect size (95% CI)	*P* for interaction
Sex			0.8870
Male	236	1.03 (1.00, 1.05)	
Female	155	1.02 (0.99, 1.05)	
Age			0.0436
<60	216	1.05 (1.02, 1.09)	
≥60	175	1.00 (0.97, 1.04)	
Respiratory failure			0.0319
Yes	87	1.00 (0.97, 1.03)	
No	304	1.05 (1.02, 1.08)	
Sepsis			0.0603
Yes	69	1.02 (1.00, 1.04)	
No	322	1.08 (1.01, 1.15)	
Glucocorticoid			0.0195
Yes	159	0.99 (0.96, 1.03)	
No	232	1.05 (1.02, 1.08)	
Tacrolimus			0.0677
Yes	143	0.99 (0.95, 1.04)	
No	248	1.04 (1.01, 1.08)	
Mycophenolate			0.0898
Yes	113	1.07 (1.01, 1.13)	
No	278	1.02 (0.99, 1.05)	

## Data Availability

The data used to support the findings of this study are available from Zuoan Qin from the second people's Hospital of Changde City, Hunan Province upon request.
